The article "Assessing the Efficacy of the Early Rehabilitation Pathway in Combination with Morita Therapy after Hip and Knee Arthroplasty" was published in 2022. Journal: J Healthc Eng.

# Assessing the Efficacy of the Early Rehabilitation Pathway in Combination with Morita Therapy after Hip and Knee Arthroplasty

**DOI:** 10.1155/2022/4285197

**Published:** 2022-03-24

**Authors:** Xin Yi, Jong Hak Lee, Xiaogui Yu, Guoliang Yi, Ho Seong Lee

**Affiliations:** ^1^Department of Kinesiologic Medical Science, Graduate School, Dankook University, Cheonan, Republic of Korea; ^2^The First Affiliated Hospital, Department of Pain, Hengyang Medical School, University of South China, Hengyang 421001, China; ^3^Institute of Medical-Sports, Dankook University, Yongin, Republic of Korea; ^4^The First Affiliated Hospital, Operating Room, Hengyang Medical School, University of South China, Hengyang 421001, China; ^5^The First Affiliated Hospital, Department of Orthopedics, Hengyang Medical School, University of South China, Hengyang 421001, China

## Abstract

Total hip arthroplasty (THA) and total knee arthroplasty (TKA) are effective methods for the treatment of end-stage osteoarthritis. Furthermore, rehabilitation training and psychological interventions play significant roles in the recovery of hip and knee joint function after THA and TKA. A total of 46 patients who received hip replacement and knee replacement are equally divided into two groups, with the control group being prescribed routine rehabilitation intervention and the observation group prescribed an early rehabilitation pathway with Morita therapy intervention. According to the results, the observation group displayed a significantly decreased incidence of deep venous thrombosis, while simultaneously reducing the recovery time of lower limb function (*P* < 0.05), including straight leg raising time, walking time, and vertical knee flexion time. In addition, the treatment program demonstrates a significant ability to improve the joint function score, pain score, quality of life score, and range of motion score (*P* < 0.05). Moreover, serum D-dimer, fibrin degradation products (FDP), and femoral vein blood flow peak also are significantly reduced (*P* < 0.05). Therefore, we have determined that an early rehabilitation pathway combined with Morita therapy can effectively reduce stress pain, improve the recovery process of joint motor function, and reduce the incidence of thrombosis. However, an increased sample size would facilitate the confirmation of the safety and efficacy of the program. In addition, the overall financial expenditure and feasibility of the treatment need to be considered.

## 1. Introduction

Total knee arthroplasty (TKA) and total hip arthroplasty (THA) are commonly employed in the clinical treatment of end-stage knee and hip disorders, and they frequently exhibit numerous therapeutic benefits [1]. However, deep venous thrombosis (DVT) is regarded as one of the most serious complications that can occur after total hip and knee arthroplasty, only secondary to the threat of a pulmonary embolism, and it can be life-threatening [2]. The incidence of DVT occurring after total hip and knee arthroplasty is recorded at 40–80% [3]. Therefore, the prevention of DVT after total hip and knee arthroplasty cannot be ignored. Slow blood flow, vascular injury, and hypercoagulability are the primary causes of DVT. The incidence of DVT after total hip and knee arthroplasty is commonly related to the incidence of intraoperative injury, the operative use of a tourniquet and bone cement, postoperative bed rest, and the patients' age [4]. In addition, the prevalence of DVT transpiring after total hip and knee arthroplasty generally occurred within 2 weeks postsurgery, with a recorded peak incidence ensuing at the 1 week time point postsurgery. Therefore, it is vitally important to initiate active and systematic prevention and intervention measures after operation to ensure an improved patient outcome that negates the risk of DVT.

The article "Assessing the Efficacy of the Early Rehabilitation Pathway in Combination with Morita Therapy after Hip and Knee Arthroplasty" was published in 2022. Journal: J Healthc Eng.

As a result of postoperative pain and psychological problems, many patients are unable to get out of bed early or engage in functional exercise, which not only prolongs the length of hospital stay and aggravates the economic burden but also produces greater mental pressure and physical pain [5]. Studies have confirmed that implementation of a scientifically ratified rehabilitation program can not only reduce the physical and mental pain of patients after surgery but also relieve the stress response produced as a result of surgery, which is conducive to the repair of tissue trauma, whilst simultaneously reducing the incidence of complications such as pressure sores, prolapse pneumonia, and deep vein thrombosis [6, 7].

It is understood that both early active and passive functional exercise after hip and knee arthroplasty can improve the rehabilitation effect on joint function [8]. The implementation of early rehabilitation training can facilitate an enhancement of lower limb exercise, prevent venous wall damage, and effectively avoid the formation of deep venous thrombosis in patients after hip and knee arthroplasty [9]. It is particularly important to execute gradual functional exercise in early rehabilitation activities based on the characteristics of the patients' condition and their pain status.

Morita therapy is a complex type of psychological intervention, which demonstrates an exceptional ability to produce significant therapeutic effects in the treatment of schizophrenia, anxiety disorder, and obsessive-compulsive disorder [10]. Improving a patients' bad mood may facilitate an enhanced positive effect on treatment and recovery. A previous study ascertained that the scores of physical functions, role function, emotional function, cognitive function, social function, and overall health status of patients are significantly improved after Morita treatment, which is of great significance for the overall rehabilitation process because it reduces stress pain, improves the recovery process of joint motor function, and reduces the chance of thrombosis [11].

The article "Assessing the Efficacy of the Early Rehabilitation Pathway in Combination with Morita Therapy after Hip and Knee Arthroplasty" was published in 2022. Journal: J Healthc Eng.

This study will explore the effect of an early rehabilitation pathway in combination with Morita therapy on the incidence of deep venous thrombosis, treatment time, joint function, pain score and quality of daily life, as well as serum D-dimer, FDP, and peak blood flow of the common femoral vein in patients after hip and knee replacement surgery [12–16].

## 2. The Research Data and Methods

The research data are obtained from a total of 46 patients who underwent hip and knee arthroplasty in the hospital. The comparison of demographic data is recorded, as given in Table 1.

The control group is the prescribed routine rehabilitation intervention. Control group patients received standard subcutaneous injections of low molecular weight heparin 12 hours after operation. The temperature, colour, and elasticity of the skin, whether the affected limb is swollen or numb, and the plane circumference of the affected limb are measured. The patency of drainage tubes and the character, colour, and quantity of drainage are also stringently observed and recorded. After waking up from anaesthesia, the patients are guided to conduct ankle flexion, back ankle extension, and quadriceps ankle contraction exercises, gradually using a machine for knee or hip passive flexion and extension and progressively increasing the angle, time, and frequency of joint activity.

The observation group is prescribed an early rehabilitation pathway. On the first day after operation, the limb function, general condition, and wound tension are evaluated. After the patient returned to the ward, the affected limb is immediately elevated, and an ice bag is used as a local cold compress, 30 min/time, with an interval of 1 h. After operation, the patients' physical signs are recorded as stable. On the first day after the operation, limb joint stretching exercises, ankle immobilization, and supine and flexion exercises are executed for a duration of 5–10 minutes once every 2 hours. During the functional exercise, the large dressing for the wound is removed, and the training intensity is gradually increased to maintain good muscle tension. Specifically, the patient's maximal endurance of pain is regarded as the appropriate intensity for training, with the patient being trained to move with stability on the floor. From the 2nd to the 7th day after operation, functional exercise gradually changed from lying to sitting, from sitting to standing, from standing to walking, and finally autonomous walking. At this stage, the primary exercise is aimed at restoring the range of motion of joints. From 6 to 8 weeks postsurgery, active knee extension training, hip joint training, and quadriceps training commenced. For patients with tibia tubercle injury and fixation during operation, active knee extension exercises are prescribed 8 weeks postsurgery. Those with meniscus injury are required to perform exercise after removing the plaster. It is strictly forbidden to walk with weight on the affected limb. At 8 weeks after operation, X-ray or CT scan is used to assess the union of joint fracture. For a severe fracture, with the help of double crutches, 50% weight is gradually loaded, and all the patients are self-weight loaded after 12–14 weeks.

The article "Assessing the Efficacy of the Early Rehabilitation Pathway in Combination with Morita Therapy after Hip and Knee Arthroplasty" was published in 2022. Journal: J Healthc Eng.

Morita therapy intervention is conducted under the direction of a certified rehabilitation therapist. Doctors and patients are encouraged to understand each other. Doctors conduct psychological evaluation of patients, guide patients to articulate their symptoms, and attempt to reduce the rejection and confrontation of symptoms. The concept of letting nature take its course to help patients accept symptoms and emotions and do what they feel they can about their individual symptoms is applied. Doctors should assist patients in shifting their attention to diseases, leading patients to experience the feeling of living like healthy people, carrying out relaxation training, and continuing training to maintain a curative effect.

This score includes measurements pertaining to pain, function, range of motion, and deformity. It is comprised of 44 points of pain and 47 points of function, including gait evaluation and function evaluation. Gait evaluation included claudication (0–11), walking distance (0–11), and use of assistive devices (0–11). The total score ≥90 is considered excellent, 80–89 is good, 70–79 is medium, and ≤69 is poor.

The VAS score can quantify abstract pain sensations into a measurable and comparative evaluation index. The concept of VAS is to add 10 scales to a 10 cm long ruler. “0” means no pain at all, and “10” means unbearable pain. The patient should point out the scale on the ruler that can best describe his/her individual pain feeling.

The Barthel index (BI) score is used to evaluate patients' daily activities, including eating, bathing, decorating, dressing, controlling defecation, controlling urination, going to the toilet, moving to the bed and chair, walking on flat ground, and going up and down stairs, encompassing a total score of 0–100.

The article "Assessing the Efficacy of the Early Rehabilitation Pathway in Combination with Morita Therapy after Hip and Knee Arthroplasty" was published in 2022. Journal: J Healthc Eng.

This score is used to evaluate the active and passive flexion and extension function. Enzyme-linked immunoturbidimetry is used to detect the D-dimer, and latex immunoturbidimetry is used to detect the FDP. The colour Doppler ultrasound of the lower limbs is performed 14 days after operation to measure the peak value of femoral vein blood flow.

The SAS scale is compiled by William W. K. Zung, consisting of 20 items and 4 grades (1–4/item). SPSS 21.0 statistical software is utilised for data analysis. The average ± standard deviation is used to express straight leg raising time, walking time, vertical knee flexion time, Harris score, ROM, VAS pain score, Barthel index, D-dimer, FDP and peak femoral venous blood flow, SAS, and SDS values. The above data are analysed by a *t*-test. The incidence of DVT is expressed as *n* (%), and a chi-square F test is used for comparison. A difference with a *P* value less than 0.05 is considered statistically significant (*P* < 0.05).

## 3. The Experimental Result

As given in Table 2, the incidence of DVT is significantly lower in the observation group than that in the control group (*P* < 0.05). Table 2 provides the comparison of the incidence of deep venous thrombosis between the groups.

The early rehabilitation pathway combined with Morita therapy can reduce the treatment time. The straight leg raising time, walking time, and vertical knee flexion time of the observation group are also significantly reduced, as given in Table 3.

The early rehabilitation pathway combined with Morita therapy can promote the rehabilitation of joint function, reduce pain, and improve the quality of daily life. The joint function score, pain score, quality of daily life, and range of motion of the observation group are significantly improved, as given in Table 4.

The early rehabilitation pathway combined with Morita therapy can reduce serum D-dimer, FDP, and the peak value of femoral vein blood flow, as given in Table 5. Table 5 provides serum D-dimer, FDP, and peak values of femoral vein blood flow.

The early rehabilitation pathway combined with Morita therapy can improve negative emotions and reduce psychological stress.  Table 6 provides the self-rating anxiety scale (SAS) and self-rating depression scale (SDS).

The scores of anxiety (SAS) and depression (SDS) in the observation group are significantly lower than those in the control group, as given in Table 6.

## 4. The Clinical Result Analysis

As previously mentioned, DVT is one of the most dangerous complications that can occur after hip and knee arthroplasty, and appropriate rehabilitation should be aimed at reducing the incidence of DVT. In our study, the occurrence of DVT in the observation group is recorded as only 1/4 of that in the control group, with this drastic reduction being of clear statistical significance (*P* < 0.05). In addition to this value, three other indicators are statistically significant, including serum D-dimer, FDP, and peak values of femoral vein blood flow, all of which are indicative of the likelihood and tendency of ensuing thrombosis. Serum D-dimer and FDP are both frequently used tools in clinical examination to evaluate patients in a hypercoagulable state or who may be threatened by thrombosis. The decrease of these two indicators indicates that the possibility of thrombosis is also correspondingly reduced. On the other hand, femoral vein blood flow, in comparison to the other two indicators designed to predict the likelihood and tendency of thrombosis, this indicator attempted to reveal why the observation group is less likely to experience clotting.

The article "Assessing the Efficacy of the Early Rehabilitation Pathway in Combination with Morita Therapy after Hip and Knee Arthroplasty" was published in 2022. Journal: J Healthc Eng.

The observation group underwent rehabilitation training at an earlier time, with more careful and gradual training in all aspects: lying to sitting and finally standing. The early rehabilitation pathway training is not aimed at initiating ordinary rehabilitation training in advance nor at blindly increasing the training content, but is rather directed at carrying out targeted and personalized training for different recovery states. In addition, those targeted exercises have demonstrated satisfactory effects as observed in the results relating to the improvement of straight leg raising time, walking time, and vertical knee flexion time, which are all demonstrated to have statistical significance (*P* < 0.05) and which all effectively reflected the quality of recovery and the function of the lower limbs. These specific rehabilitation exercises, while assisting the recovery process, also facilitated increased blood flow of the femoral vein in this study, which effectively reduces the threat of postoperative complications.

The advantage of early rehabilitation pathway training impacts not only the speed of rehabilitation but also the quality. The four scores in this study all reflect the quality of recovery after hip and knee arthroplasty. The Harris score reflects the recovery degree after hip replacement, and the VAS pain score reflects the pain experienced by patients during recovery. Excessive pain will inevitably lead to the reduction of training compliance, which indirectly affects the recovery process in conjunction with the quality of life after recovery. Improvement of the VAS pain score causes increased patient training compliance, which ultimately contributes to the improvement of other scores, and these scores are combined to certify the advantage of an early rehabilitation pathway in recovery from hip and knee arthroplasty.

The article "Assessing the Efficacy of the Early Rehabilitation Pathway in Combination with Morita Therapy after Hip and Knee Arthroplasty" was published in 2022. Journal: J Healthc Eng.

Furthermore, this study also suggests that significant improvement in the overall recovery effect is also positively influenced by the implementation of Morita therapy, which is largely concerned with the psychological treatment of depression and anxiety. Although positive psychological responses have been shown to promote postoperative recovery in general, no studies have directly demonstrated the acceleration of recovery from major surgery with Morita therapy. This study is the first to apply Morita therapy to improve the mental state of patients in postoperative rehabilitation after major surgery, and obviously, both anxiety and depression scores improved significantly (*P* < 0.05) in the observation group that received Morita therapy.

## 5. Conclusion

The application of an early rehabilitation pathway in combination with Morita therapy can significantly reduce the incidence of deep vein thrombosis, shorten the treatment time, promote the rehabilitation of joint function, relieve pain symptoms, relieve anxiety and depression, and improve the quality of daily life. However, most clinicians and patients have not yet realized the fundamental importance of rehabilitation and psychological intervention after hip and knee arthroplasty, and more data are required to substantiate the underlying mechanisms and confirm the therapeutic efficacy of these treatments.

## Figures and Tables

**Table 1:** Demographic data of the two cohorts: hip replacements and knee replacements.

Group	Gender		Age (years)
	Male	Female	
Control group (*n* = 23)	10	13	67.54 ± 1.29
Observation group (*n* = 23)	9	14	68.27 ± 1.34
*t*/*F*	15.235	20.685	8.43
*P*	0.96	0.93	0.82

**Table 2:** Comparison of the incidence of deep venous thrombosis between the groups.

Group	Incidence of deep venous thrombosis (*n*, %)
Control group (*n* = 23)	8, 34.8
Observation group (*n* = 23)	2, 8.7
*X* ^2^	4.511
*P*	0.034

**Table 3:** Functional recovery of the lower limbs.

Group	Straight leg raising time (d)	Walking time (d)	Vertical knee flexion time (d)
Control group (*n* = 23)	1.76 ± 0.51	2.48 ± 0.67	2.19 ± 0.55
Observation group (*n* = 23)	1.34 ± 0.21	2.03 ± 0.55	1.68 ± 0.38
*t*	3.807	2.596	3.814
*P*	<0.01	0.013	<0.01

**Table 4:** Assessment of joint function, pain, and quality of life.

Group	Harris score	VAS pain score	Life quality score	Range of motion (ROM)
Control group (*n* = 23)	80.11 ± 8.42	1.51 ± 0.32	71.22 ± 5.12	101.21 ± 8.42
Observation group (*n* = 23)	88.12 ± 10.32	1.11 ± 0.25	79.22 ± 6.25	108.12 ± 10.33
*t*	4.253	6.965	6.914	3.667
*P*	<0.01	<0.01	<0.01	<0.01

The article "Assessing the Efficacy of the Early Rehabilitation Pathway in Combination with Morita Therapy after Hip and Knee Arthroplasty" was published in 2022. Journal: J Healthc Eng.

**Table 5:** Serum D-dimer, FDP and Peak values of femoral vein blood flow.

Group	serum D-dimer (mg/L)	FDP (ug/L)	Peak blood flow of common femoral vein (cm/s)
Control group (*n* = 23)	0.34 ± 0.09	11.6 ± 2.4	19 ± 4
Observation group (*n* = 23)	0.29 ± 0.09	10.5 ± 2.1	21 ± 4
*t*	5.364	7.076	7.025
*P*	<0.01	<0.01	<0.01

**Table 6:** Self-rating anxiety scale (SAS) and self-rating depression scale (SDS).

Group	SAS	SDS
Control group (*n* = 23)	54 ± 3.1	53 ± 2.4
Observation group (*n* = 23)	42 ± 1.3	40 ± 1.7
*T*	47.218	46.312
*P*	<0.01	<0.01

## Data Availability

The data used to support the findings of this study are available from the corresponding author upon request.
